The article "An Efficient Adaptive Salp Swarm Algorithm Using Type II Fuzzy Entropy for Multilevel Thresholding Image Segmentation" was published in 2022. Journal: Comput Math Methods Med.

# An Efficient Adaptive Salp Swarm Algorithm Using Type II Fuzzy Entropy for Multilevel Thresholding Image Segmentation

**DOI:** 10.1155/2022/2794326

**Published:** 2022-01-29

**Authors:** Shubham Mahajan, Nitin Mittal, Rohit Salgotra, Mehedi Masud, Hesham A. Alhumyani, Amit Kant Pandit

**Affiliations:** ^1^School of Electronics & Communication, Shri Mata Vaishno Devi University, Katra-182320, India; ^2^Department of Electronics & Communication Engineering, Chandigarh University, Mohali, India; ^3^School of Mechanical Engineering, Iby & Aladar Fleishman Faculty of Engineering Tel Aviv University, Israel; ^4^Department of Computer Science, College of Computers and Information Technology, Taif University, P.O. Box 11099, Taif 21944, Saudi Arabia; ^5^Department of Computer Engineering, College of Computers and Information Technology, Taif University, P.O. Box 11099, Taif 21944, Saudi Arabia

## Abstract

Salp swarm algorithm (SSA) is an innovative contribution to smart swarm algorithms and has shown its utility in a wide range of research domains. While it is an efficient algorithm, it is noted that SSA suffers from several issues, including weak exploitation, convergence, and unstable exploitation and exploration. To overcome these, an improved SSA called as adaptive salp swarm algorithm (ASSA) was proposed. Thresholding is among the most effective image segmentation methods in which the objective function is described in relation of threshold values and their position in the histogram. Only if one threshold is assumed, a segmented image of two groups is obtained. But on other side, several groups in the output image are generated with multilevel thresholds. The methods proposed by authors previously were traditional measures to identify objective functions. However, the basic challenge with thresholding methods is defining the threshold numbers that the individual must choose. In this paper, ASSA, along with type II fuzzy entropy, is proposed. The technique presented is examined in context with multilevel image thresholding, specifically with ASSA. For this reason, the proposed method is tested using various images simultaneously with histograms. For evaluating the performance efficiency of the proposed method, the results are compared, and robustness is tested with the efficiency of the proposed method to multilevel segmentation of image; numerous images are utilized arbitrarily from datasets.

## 1. Introduction

Nature-inspired methods are applied in most engineering research problems because of their linear nature, easy implementation, and randomization dependent on population. They are mainly classified into two major types: swarm intelligence (SI) and evolutionary algorithms (EAs). EAs are methods that work on optimization of the research problem, e.g., differential evolution (DE) [1], genetic algorithm (GA) [2], and ant lion optimizer (ALO) [3]. SI is dependent on the swarming nature of various species, e.g., dragonfly algorithm (DA) [4], firefly algorithm (FA) [5], gray wolf optimization (GWO), bat algorithm (BA) [6, 7], and particle swarm optimization (PSO) [8–10].

The article "An Efficient Adaptive Salp Swarm Algorithm Using Type II Fuzzy Entropy for Multilevel Thresholding Image Segmentation" was published in 2022. Journal: Comput Math Methods Med.

Segmentation is aimed at distinguishing several essential parts that define objects. Segmentation, a challenging step in image processing, plays a key role in detecting objects and pattern recognition [11]. It is necessary to develop an image segmentation algorithm that does not require human intervention and minimal computational resources. The solution to the problem previously proposed relies on *C* and *K*-means clustering algorithms [12, 13]. But the cluster number computation was its key drawback, along with the fact that the system's computing complexity increased exponentially.

Furthermore, histogram-based thresholding has provided the solution to the image segmentation, where the number of thresholds (th) and histograms would be used together with objective function. The two broadly employed objective functions proposed presently are the Kapur criteria for entropy [14] and Otsu class variance [15]. The above-stated methods are useful but also increase the computational cost when used with multilevel thresholding. Various methods of optimization have been used by researchers from a while to solve this problem.

Some drawbacks of Kanpur entropy were overcome in firefly optimization algorithm (FOA) This approach recreates the behavior of fireflies and bioluminescent interaction processes in nature [5]. Horng also proposed the use of honey bee mating optimization (HBO) in multilevel image thresholds with Kapur's entropy (KE) [16]. The problem of class variance function and the optimization of the entropy criterion in multilevel thresholding was overcome by the bacterial foraging algorithm (BFA) [17, 18] and harmony search optimization system (HSO) [19], but Tuba and Brajevic preferred the use of FOA [11] and cuckoo search (CS) [6]. The CS system and Kapur entropy segmentation of satellite images were used. Otsu's approach was tested with the firefly algorithm (FA) [20] for multilevel image thresholds. Tuba and Alihodzic [21] used a bat algorithm (BA) with Otsu and Kapur in multilevel image thresholds. Effective results were obtained when the Tsallis, Kapur, and Otsu methods were optimized using the modified artificial bee colony system for multilevel thresholding images [21]. Subsequently, multilevel picture thresholding was used for the gray wolf optimization process (GWO); an objective function was dependent on Otsu's class variance method [22] and Kapur's entropy. Animal migration optimization (AMA) and social spider (SSA) algorithm were used to optimize class variance for thresholding multilevel images using Otsu class variance methods and Kapur entropy [23, 24]. Interdependence has been reduced using an adaptive balance optimizer (AEO) with a multilevel threshold [25]. Additional segmentation of images was carried out using the exchange market optimization (EMO) approach with a minimum cross-entropy threshold [26]. Elaziz et al. [27] used a hyperheuristic approach to threshold multilevel images by optimizing class variance to address the drawback of a metaheuristic method. While optimization approaches used so far have been effective with the user-defined threshold value, we have not achieved a completely programmed segmentation method.

The article "An Efficient Adaptive Salp Swarm Algorithm Using Type II Fuzzy Entropy for Multilevel Thresholding Image Segmentation" was published in 2022. Journal: Comput Math Methods Med.

When multilevel thresholding, a separate method is used along with peak detection, which relies on the information in the histogram, so the objective function where the cluster center is the peak value of the histogram and the valley is the upper and lower limit of the cluster determined by the intensity level of the histogram, it can be said that the pixel intensity between successive valleys is taken as a cluster in the picture [28, 29]. Methods for detecting peaks in the histogram were proposed by Tsai, where Gaussian kernel smoothing was used to eliminate variable peaks and valleys [30], which are the best methods for finding two peaks not fail to detect more than two peaks in the image.

In this article, a novel technique of ASSA along with thresholding methods is proposed for image segmentation, which is an area of research with high accuracy in segmentation. It is practically validated by testing the accuracy of outputs and computational time taken by many other existing, state-of-the-art algorithms like GA [2], PSO [8], FPA [5], BA [6, 7], CS [9], DE [1], and MPA [10].

The main contributions of this paper are as follows:

1. The use of ASSA for optimum multilevel thresholding with TII-FE: experiment results indicate that ASSA produces better results than PFA-, DE-, PPA-, PSO-, MPA-, and HPFPPA-D-dependent techniques
2. The computation of multilevel thresholding is significantly reduced by using ASSA-based TII-FE

The paper is planned as follows: a detailed introduction of thresholding in multilevel images is discussed in Section 2. The fundamentals of ASSA are described in Section 3. Results are detailed in Section 4. At last, in Section 5, the conclusion and future scope of the work is discussed.

## 2. Thresholding in Multilevel Images

Optimal thresholding techniques [11] are employed in image processing to determine thresholds, so the clusters formed on histograms follow the target objectives. The probability of *i*^th^ the gray level is

(1) $$\begin{array}{c} p_{i}=\frac{h_{i}}{M\times N}, \end{array}$$

where the range of gray level is {0, 1, 2, 3, 4, 5 ⋯ ⋯⋯⋯⋯.*L* − 1}, *M* × *N* is the image dimension, and *h*_*i*_ is the no. of pixels with gray level *i*, 0 ≤ *i* ≤ (*L* − 1).

The article "An Efficient Adaptive Salp Swarm Algorithm Using Type II Fuzzy Entropy for Multilevel Thresholding Image Segmentation" was published in 2022. Journal: Comput Math Methods Med.

Let *m* be the no. of thresholds present; then, *t*_1_, *t*_2_, *t*_3_, *t*_4_, ⋯⋯⋯..*t*_*m*_ and if we break it in *m* classes, then

(2) $$\begin{array}{c} C_{0}=\left\{0,\cdots \cdots .t_{1}-1\right\},\\ C_{1}=\left\{t_{1},\cdots \cdots .t_{2}-1\right\},\\ C_{2}=\left\{t_{2},\cdots \cdots .t_{3}-1\right\},\\ C_{3}=\left\{t_{3},\cdots \cdots .t_{4}-1\right\},\\ :\\ C_{m}=\left\{t_{m},\cdots \cdots .L-1\right\}. \end{array}$$

Optimal thresholds are achieved by increasing the objective function that is based on specified parameters of thresholds. The most widely applied optimum thresholding techniques are Otsu's and Kapur's methods [14, 15]. The objective function in bilevel thresholding is selected as per Kapur's approach:

(3) $$\begin{array}{c} J\left(t_{1}\right)=H_{0}+H_{1}, \end{array}$$

where

(4) $$\begin{array}{c} H_{0}=-\overset{t_{1}-1}{\underset{i=0}{\sum }}\frac{p_{i}}{\omega_{0}}\ln\frac{p_{i}}{\omega_{0}},\\ \omega_{0}=\overset{t_{1}-1}{\underset{i=0}{\sum }}p_{i},\\ H_{1}=-\overset{L-1}{\underset{i=t_{1}}{\sum }}\frac{p_{i}}{\omega_{1}}\ln\frac{p_{i}}{\omega_{1}},\\ \omega_{1}=\overset{L-1}{\underset{i=t_{1}}{\sum }}p_{i}. \end{array}$$

*H*_0_&*H*_1_ are partial entropies of histogram.

*t*_1_ is the gray level, which increases objective function in Equation (3).

Now, by Otsu's method, it is defined

(5) $$\begin{array}{c} J\left(t_{1}\right)=\sigma_{0}+\sigma_{1}, \end{array}$$

where

(6) $$\begin{array}{c} \sigma_{0}=\omega_{0}\;{\left(\mu_{0}-\mu_{T}\right)}^{2},\\ \sigma_{1}=\omega_{1}\;{\left(\mu_{1}-\mu_{T}\right)}^{2},\\ \omega_{0}=\overset{t_{1}-1}{\underset{i=0}{\sum }}p_{i},\\ \mu_{0}=\overset{t_{1}-1}{\underset{i=0}{\sum }}\frac{{ip}_{i}}{\omega_{0}},\\ \omega_{1}=\overset{L-1}{\underset{i=t_{1}}{\sum }}p_{i},\\ \mu_{1}=\overset{L-1}{\underset{i=t_{1}}{\sum }}\frac{{ip}_{i}}{\omega_{0}},\\ \mu_{T}=\overset{L-1}{\underset{i=t_{1}}{\sum }}ip_{i}. \end{array}$$

Therefore, *ω*_0_*μ*_0_ + *ω*_1_*μ*_1_ = *μ*_*T*_ and *ω*_0_+*ω*_1_ = 1 and *μ*_*T*_ is the mean intensity.

Thresholding for multilevel images can be increased by Kapur's entropy; *m*-dimensional optimization problem is optimal [11] in which *m*-optimal thresholds (*t*_1_, *t*_2_, *t*_3_, *t*_4_, ⋯⋯⋯..*t*_*m*_) are examined by increasing objective function:

(7) $$\begin{array}{c} J\left(t_{1},t_{2},t_{3},t_{4},\cdots \cdots \cdots ..t_{m}\right)=H_{0}+H_{1}+H_{2}+H_{3}+H_{4}+\cdots \cdots \cdots .+H_{m}, \end{array}$$

where

(8) $$\begin{array}{c} H_{0}=-\overset{t_{1}-1}{\underset{i=0}{\sum }}\frac{p_{i}}{\omega_{0}}\ln\frac{p_{i}}{\omega_{0}},\\ \omega_{0}=\overset{t_{1}-1}{\underset{i=0}{\sum }}p_{i},\\ H_{1}=-\overset{t_{2}-1}{\underset{i=t_{1}}{\sum }}\frac{p_{i}}{\omega_{1}}\ln\frac{p_{i}}{\omega_{1}},\\ \omega_{1}=\overset{t_{2}-1}{\underset{i=t_{1}}{\sum }}p_{i},\\ :\\ H_{m}=-\overset{L-1}{\underset{i=t_{m}}{\sum }}\frac{p_{i}}{\omega_{m}}\ln\frac{p_{i}}{\omega_{m}},\\ \omega_{m}=\overset{L-1}{\underset{i=t_{m}}{\sum }}p_{i}. \end{array}$$

Now, by Otsu's method as in Equation (5), it is defined

(9) $$\begin{array}{c} J\left(t_{1},t_{2},t_{3},t_{4},\cdots \cdots \cdots ..t_{m}\right)=\sigma_{0}+\sigma_{1}+\sigma_{2}+\sigma_{3}+\sigma_{4}+\cdots \cdots \cdots .+\sigma_{m},\\ \sigma_{0}=\omega_{0}\;{\left(\mu_{0}-\mu_{T}\right)}^{2},\\ \sigma_{1}=\omega_{1}\;{\left(\mu_{1}-\mu_{T}\right)}^{2},\\ :\\ \sigma_{m}=\omega_{m}\;{\left(\mu_{m}-\mu_{T}\right)}^{2},\\ \omega_{0}=\overset{t_{1}-1}{\underset{i=0}{\sum }}p_{i},\\ \mu_{0}=\overset{t_{1}-1}{\underset{i=0}{\sum }}\frac{{ip}_{i}}{\omega_{0}},\\ \omega_{1}=\overset{t_{2}-1}{\underset{i=t_{1}}{\sum }}p_{i},\\ \mu_{1}=\overset{t_{2}-1}{\underset{i=t_{1}}{\sum }}\frac{{ip}_{i}}{\omega_{0}},\\ :\\ \omega_{m}=\overset{L-1}{\underset{i=t_{m}}{\sum }}p_{i},\\ \mu_{m}=\overset{L-1}{\underset{i=t_{m}}{\sum }}\frac{{ip}_{i}}{\omega_{m}}. \end{array}$$

The value of thresholds is *t*_1_ < *t*_2_ < *t*_3_ < *t*_4_, ⋯⋯⋯<*t*_*m*_ in both methods.

The article "An Efficient Adaptive Salp Swarm Algorithm Using Type II Fuzzy Entropy for Multilevel Thresholding Image Segmentation" was published in 2022. Journal: Comput Math Methods Med.

### 2.1. Multilevel Thresholding with Fuzzy Type II Sets

The segmentation obtained by multilevel thresholding methods works by grouping pixels based on intensity values to facilitate image analysis. The segmentation criteria can be divided into two types: parametric and nonparametric. In comparison to nonparametric parameters, metric methodologies are considered to produce more computational weight. As a result, nonparametric techniques are often preferred due to their intensity and simplicity, maximum entropy, and the most well-known between-class variance.

Researchers paid close attention to entropy-based data utilized to separate the image's histogram. To start with, the data hypothesis allowed us to apply Shannon's entropy to the thresholding problem [31]. Regarding this trend, several different methodologies, such as Tsallis entropy [32], Renyi's entropy [33], cross-entropy [34], and finally a fuzzy entropy-based approximation [35], were suggested. Segments are used to remove artifacts from images.

The article "An Efficient Adaptive Salp Swarm Algorithm Using Type II Fuzzy Entropy for Multilevel Thresholding Image Segmentation" was published in 2022. Journal: Comput Math Methods Med.

Moreover, when many edges are used, most entropy-based criteria will suffer from the negative effects of high complexity. Tao et al. [36] introduced a fuzzy entropy-based method to improve Zhao's [37] work. An image is thresholded using histogram segments with specified fuzzy membership values; these segments are used to eliminate objects in an image.

#### 2.1.1. Different Fuzzy Type II Sets

Type I fuzzy, with finite set *X* = (*x*_1_, *x*_2_, ⋯⋯, *x*_*n*_), is defined in

(10) $$\begin{array}{c} A=\left\{x,\mu_{A}\left(x\right)\;|\;x\in X,0\leq \mu_{A}\left(x\right)\leq 1\right\}, \end{array}$$

where *μ*_*A*_ is the membership function.

For dealing with vulnerability, a number of membership values are used in fuzzy type II sets rather than value as in

(11) $$\begin{array}{c} A=\left\{x\mu_{A}^{\text{high}}\left(x\right),\mu_{A}^{\text{low}}\left(x\right)\;|\;x\in X,0\leq \mu_{A}^{\text{high}}\left(x\right),\mu_{A}^{\text{low}}\left(x\right)\leq 1\right\}, \end{array}$$

where *μ*_*A*_^high^(*x*) and *μ*_*A*_^low^(*x*) are the upper and lower membership functions.

#### 2.1.2. Image Segmentation with Fuzzy Type II

Thresholding is the simplest method for segmenting an image. Thresholding is as simple as using a threshold (th) value and adding it to a histogram until an optimal condition is reached. Equation (12) describes the thresholding method using a histogram.

(12) $$\begin{array}{c} I_{s}\left(r,c\right)=\left\{\begin{array}{c} I_{Gr}\left(r,c\right)\text{ if }I_{\text{Gr}}\left(r,c\right)\leq {\text{th}}_{1},\\ {\text{th}}_{k-1}\text{ if }{\text{th}}_{k-1}<I_{\text{Gr}}\left(r,c\right)\leq {\text{th}}_{k},k=2,3,\cdots .nt,\\ I_{\text{Gr}}\left(r,c\right)\text{ if }I_{\text{Gr}}\left(r,c\right)>{\text{th}}_{nt}, \end{array}\right. \end{array}$$

where *I*_*s*_(*r*, *c*) is the segmented image with gray value, *I*_Gr_(*r*, *c*) is the original image with gray value, and (*r*, *c*) is the position of pixels.

## 3. Adaptive Salp Swarm Algorithm

### 3.1. Salp Swarm Algorithm

The SSA method is SI inspired by navigation and foraging activity of salps present in oceans [38]. Body configuration of salps is very closely linked to jellyfish present in oceans and practices the same technique to step forth and pump water across their bodies. SSA is ultimately inspired by the swarming action of the salps under which the swarm of the salps produces a chain of salps. The leader salp is present in front, and the rest who follow the leader are known as followers. The position of salps in search space is determined by the presence of food source *S* and leader's position by

(13) $$\begin{array}{c} Y_{j}^{i}=\left\{\begin{array}{c} S_{j}+c_{1}\left(\left({\text{ub}}_{j}-{\text{lb}}_{j}\right)c_{2}+{\text{lb}}_{j}\right)C_{3}\geq 0,\\ S_{j}-c_{1}\left(\left({\text{ub}}_{j}-{\text{lb}}_{j}\right)c_{2}+{\text{lb}}_{j}\right)C_{3}\leq 0, \end{array}\right. \end{array}$$

where *Y*_*j*_^*i*^ is the leader/first salp, *S*_*j*_ is the food source at *j*^th^ dimensions, ub_*j*_ and lb_*j*_ are the upper and lower boundary, *c*_1_, *c*_2_, *c*_3_ ⋯ ⋯. are random values.

The article "An Efficient Adaptive Salp Swarm Algorithm Using Type II Fuzzy Entropy for Multilevel Thresholding Image Segmentation" was published in 2022. Journal: Comput Math Methods Med.

Balance between exploitation and exploration is maintained by *c*_1_ coefficient parameter, as shown in

(14) $$\begin{array}{c} c_{1}=2e^{-{\left(\frac{4i}{I}\right)}^{2}}, \end{array}$$

where *i* is the current iteration, *I* is the no. of iterations, and *c*_2_ and *c*_3_ are uniformly distributed random value coefficients in [0, 1].

The next position in *j*^th^ dimension is determined by utilizing these positions when moving in +ve&−ve∞.

Now, followers' updated position is shown in

(15) $$\begin{array}{c} Y_{j}^{k}=\frac{1}{2}{at}^{2}+v_{0}t, \end{array}$$

where *k* ≥ 2 and *Y*_*j*_^*k*^ is the *k*^th^ follower position in the *j*^th^ dimension.

(16) $$\begin{array}{c} v_{0}=\text{speed},\\ t=\text{time},\\ a=\frac{v_{\text{final}}}{v_{0}}. \end{array}$$

If we put *v*_0_ = 0 in Equation (15), then

(17) $$\begin{array}{c} Y_{j}^{k}=\frac{1}{2}\left(Y_{j}^{k}+Y_{j}^{k-1}\right), \end{array}$$

where *k* ≥ 2 and *Y*_*j*_^*k*^ is the *k*^th^ salp follower in the *j*^th^ dimension search area.

Some main disadvantages of SSA [39] are as follows:

1. The computational cost of the method increases due to usage of only one parameter of optimization. Although it is said that only parameter *c*_1_ is needed for optimum function, but there are 3 parameters *c*_1_, *c*_2_, and *c*_3_ present and defined
2. It has weak convergence and local optimization problems that need to be modified to increase efficiency and decrease computational cost
3. SSA should be adaptive to reduce the user depend parameter initialization and make it more effective and self-adaptive

### 3.2. Adaptive Salp Swarm Algorithm

To overcome the above-stated drawbacks of SSA, an ASSA was proposed.

Some major changes done to overcome drawbacks of SSA [38, 39] are as follows:

- For appropriate exploitation and exploration in SSA, a division depend concept was introduced in ASSA
- The major advantage is the inclusion of the logarithmic distributed (LD) parameter *c*_1_ in SSA. Randomized LD-dependent parameter is useful in shifting it towards the exploitation stage
- Balance b/w exploitation and exploration is improved by changing *c*_1_ in SSA to LD, which is useful in shifting it towards the exploitation stage
- The total no. of evaluation functions is reduced by reducing population size. It reduces computational complexity burden

The initialization of the algorithm starts in a fixed range and is presented in mathematical form as

(18) $$\begin{array}{c} x_{i,j}=x_{\min,j}+U\left(0,1\right)\times \left(x_{\min,j}-x_{\max,j}\right), \end{array}$$

where *x*_*i*,*j*_ is the *i*^th^ solution for the *j*^th^ dimension.

(19) $$\begin{array}{c} i=\left[1,2,3,4,\cdots \cdots ,n\right],\\ j=\left[1,2,3,4,\cdots \cdots \cdots ..,d\right]. \end{array}$$

*x*_max,*j*_ and *x*_min,*j*_ are the upper and lower limits.

The article "An Efficient Adaptive Salp Swarm Algorithm Using Type II Fuzzy Entropy for Multilevel Thresholding Image Segmentation" was published in 2022. Journal: Comput Math Methods Med.

*U*(0, 1) is the uniform rand. no. in [0, 1].

Position in ASSA is updated by modifying exploitation and exploration function of SSA, and it overall increases the performance and is presented as

(20) $$\begin{array}{c} x_{1}=x_{i}-A_{1}\left(C_{1}\cdot x_{\text{new}}-x_{i}^{t}\right),\\ x_{2}=x_{i}-A_{2}\left(C_{2}\cdot x_{\text{new}}-x_{i}^{t}\right),\\ x_{3}=x_{i}-A_{3}\left(C_{3}\cdot x_{\text{new}}-x_{i}^{t}\right),\\ x_{\text{new}}^{t+1}=\frac{x_{1}+x_{2}+x_{3}}{3},\\ x_{\text{new}}^{t+1}=x_{\text{new}}^{t}+\alpha \times L\left(\lambda \right)\left(x_{\text{best}}-x_{\text{new}}^{t}\right), \end{array}$$

where *x*_new_ is the new solution, *A*_1_, *A*_2_, *A*_3_ and *C*_1_, *C*_2_, *C*_3_ are derived from *A* = 2*a* · *r*_1_ − *a* and *C*2 · *r*_2_, *α* and *L*(*λ*) are uniformly and Levy distributed rand. no., and *r*_1_ and *r*_2_ are rand. no. distribution in [0, 1].

Step size dependent on Levy flight is

(21) $$\begin{array}{c} L\left(\lambda \right)\sim \frac{\lambda \Gamma \left(\lambda \right)\sin\left(\pi_{2}^{\lambda }\right)}{\pi }\frac{1}{s^{1+\lambda }};\left(s\gg s_{0}\gg 0\right), \end{array}$$

where *s* = (*U*/(|*V*|^1^/*λ*)) *U* ~ *N*(0, *σ*^2^).

(22) $$\begin{array}{c} V\sim N\left(0,1\right),\\ \sigma^{2}=\left\{\frac{\Gamma \left(1+\lambda \right)}{\lambda \Gamma \left[1+\lambda \right]/2}.\frac{\sin\left(\pi \lambda /2\right)}{2^{\lambda -1/2}}\right.. \end{array}$$

*λ*Γ is the gamma function.

(23) $$\begin{array}{c} \lambda =1.5. \end{array}$$

*N* is derived from Gaussian distribution with variance = *σ*^2^ and mean = 0.

Basic functions of SSA and ASSA are shown in Table 1. In the selection step, greedy selection (GS) is executed to find the proposed solution optimum or not compared with already proposed methods. For a minimization method with fitness *F*(*x*_*i*_^*t*^) with *x*_*i*_^*t*^, the solution is mathematically denoted as

(24) $$\begin{array}{c} x_{\text{new}}^{t+1}=\left\{\begin{array}{c} x_{\text{new if }F\left(x_{\text{new}}\right)<F\left(x_{i}^{t}\right)},\\ x_{i}^{t}\text{ otherwise}. \end{array}\right. \end{array}$$

In controlling parameter balance b/w exploitation and exploration is improved by changing *c*_1_ in SSA to LD, which is useful in shifting it towards the exploitation stage. In this range, upper and lower *c*_max_&*c*_min_ is [0.95 0.05] represented as

(25) $$\begin{array}{c} c_{1}=c_{\max}+\left(c_{\min}-c_{\max}\right)\times \log_{10}\left(a+\frac{10t}{t_{\max}}\right), \end{array}$$

where *c* is the weight of inertia, *a* is the rand. no. in [0, 1], and *t* and *t*_max_ are present and max. no. of iterations.

The article "An Efficient Adaptive Salp Swarm Algorithm Using Type II Fuzzy Entropy for Multilevel Thresholding Image Segmentation" was published in 2022. Journal: Comput Math Methods Med.

In population adaptation, the total no. of evaluation functions is reduced by reducing population size. It reduces computational complexity burden and is represented as

(26) $$\begin{array}{c} n\left(g+1\right)=\text{round}\left[\left(\frac{n_{\min}-n_{\max}}{{\text{FEs}}_{\max}}\right)\cdot \text{FEs}+n_{\max}\right], \end{array}$$

where FEs is the max. no. of iterations and *n*_min_ − *n*_max_ is the min. and max. population size.

## 4. Result and Discussion

For simulations, MATLAB R2020a is installed on a workstation with an Intel i5-4210 CPU running at 1.70 GHz. The ASSA technique is evaluated in conditions of image segmentation, focusing on the thresholding with fuzzy II entropy. Natural images with diverse histogram distributions are used to test the suggested method. The proposed multilevel thresholding utilizing ASSA is compared to other evolutionary algorithms like PSO, PPA, PFA, DE [3–10], and HPFPPA-D [32] on ten benchmark images with varied attributes and complexities [40]. The complete step-by-step overview and working of the proposed model are represented in Figure 1.

Because evaluated algorithms contain stochastic operators, results must be studied in a statistical framework. The results of all tests are presented in this work after 30 independent runs, with parameter values for competing algorithms listed in Table 2. Finally, the problem's dimension size is defined as 2 times total number of thresholds.

For each of the segmentation approaches, three criteria have been used to determine their quality. The peak signal-to-noise ratio (PSNR) compares the segmented and original images for similarity. The PSNR is focused on the mean squared error (MSE) of each pixel [41–42]. To compare the segmented image structures, the structural similitude index (SSIM) is used. The higher SSIM number, the better the original image segmentation [43, 44].

The ASSA's results for optimizing TII-FE for thresholding are presented and analyzed in this section.  Table 3 shows best ASSA-generated thresholds for various numbers of thresholds on the benchmark images [45, 46]. The fuzzy parameters of membership functions used for threshold level estimation are described in Table 4. Tables 4 and 5 additionally include the best results produced using PSO, HPFPPA-D, DE, PPA, and PFA for comparison.  Table 6 lists the type II fuzzy entropy values achieved by each algorithm so that performance parameters can be compared. In most circumstances, the suggested ASSA outperforms comparative techniques by obtaining solutions with higher fitness values.

The article "An Efficient Adaptive Salp Swarm Algorithm Using Type II Fuzzy Entropy for Multilevel Thresholding Image Segmentation" was published in 2022. Journal: Comput Math Methods Med.

Figure 2 shows the results of ASSA-dependent segmentation graphically. Every segmented image [47] includes a histogram image and a threshold location. It is clear to notice how the output improves as the number of thresholds increases on resultant images. For evaluating the effectiveness of evolutionary computing methods, the fitness value is not the sole criteria. The convergence curve is frequently evaluated and compared to other algorithms. Figure 2 also shows the fitness evolution of the competitive approaches for benchmark image set across 50 iterations. The graphs show that the proposed strategy converges faster than other alternatives in vast majority of situations.

Table 5 displays quality metric values to demonstrate the superior quality of the images acquired with ASSA and TII-FE than any other equivalent methodologies in the segmented images. The ASSA performs better over its peers for most of the experiments in terms of MSE metric, PSNR, and SSIM. This means that there is less noise in threshold images created in this work using the method outlined and the structures which depict the images' objects are appropriately preserved.

A new approach of image threshold based on type II entropy (TII-FE) and ASSA is presented in this paper. A number of benchmark images were used to test the performance of the proposed ASSA-based threshold method. The threshold approach is evaluated against competitive methods based on image accuracy, convergence characteristics, and segmented image quality. In terms of MSE, PSNR, and SSIM, the quality of segmented image is measured. The results show that TII-FE ASSA is an effective image thresholding approach.

## 5. Conclusion and Future Scope

This paper presents an image segmentation method of thresholding using ASSA combined with type II fuzzy entropy. ASSA's fuzzy entropy type II results are more efficient than PFA, PPA, DE, PSO, and HPFPPA-D. Optimal image thresholding is accomplished by increasing the value of entropy, which is a time-consuming process. As a result, the proposed methodology is examined and studied using several performance characteristics such as MSE, PSNR, and SSIM. The results are compared to known approaches, and the robustness and effectiveness of the proposed strategy to multilevel picture segmentation are evaluated.

The article "An Efficient Adaptive Salp Swarm Algorithm Using Type II Fuzzy Entropy for Multilevel Thresholding Image Segmentation" was published in 2022. Journal: Comput Math Methods Med.

In the future, more precise segmentation of image with less computational time can be achieved by improving the method further and comparing the same with other state-of-the-art algorithms MBO [48], IOA [49], and CASF [50], which is needed in real-time applications.

## Figures and Tables

**Figure 1:** Step-by-step working of the proposed method.

**Figure 2:** Segmented test images along with equivalent histogram and convergence plots by ASSA combined with type II fuzzy entropy for 3, 5, and 7 levels.

**Table 1:** Basic functions of SSA and ASSA.

Basic functions	SSA	ASSA
Initialization of population	Rand. no.	Decreasing adaptive population
Exploitation	Standard	Standard
Exploration	Standard	Combination of CS [6] and GWO [7]
Parameters for controlling	Rand. no.	LD w.r.t. iterations

**Table 2:** Parameter settings.

Algorithm	Parameters
PSO	NP = 10 × *D*; *D* = 2 × PR = 2 × [3, 5, 7]; *G*_max_ = 50; *W*_max_ = 0.9, *W*_min_ = 0.4, Ac1 = Ac2 = 2
DE	NP = 10 × *D*; *D* = 2 × PR = 2 × [3, 5, 7]; *G*_max_ = 50; *F* = 0.5
PPA	NP = 10 × *D*; *D* = 2 × PR = 2 × [3, 5, 7]; *G*_max_ = 50; *N*_max_ = 7
PFA	NP = 10 × *D*; *D* = 2 × PR = 2 × [3, 5, 7]; *G*_max_ = 50; *σ* = 5
HPFPPA-D	NP = 10 × *D*; *D* = 2 × PR = 2 × [3, 5, 7]; *G*_max_ = 50; *N*_max_ = 7; *σ* = 5
ASSA	NP = 10 × *D*; *D* = 2 × PR = 2 × [3, 5, 7]; *G*_max_ = 50

Here, NP is the population size, *D* is the dimension of problem, *G*_max_ is the number of iteration, *N*_max_ is the maximum number of runners, *σ* is the standard deviation, bp is the breeders' probability, and PR are different threshold levels.

**Table 3:** Thresholds achieved after applying the ASSAs and competitive algorithms to segment the set of benchmark images using TII-FE.

Im	PR	ASSA	HPFPPA-D	PSO	PFA	DE	PPA
41004	3	29 104 224	33 66 137	34 144 235	35 104 193	35 100 185	36 86 152
	5	45 86 135 167 247	34 100 135 174 233	36 78 114 181 235	35 100 136 174 232	39 78 115 158 209	35 105 151 191 236
	7	19 62 98 124 157 202	41 84 115 146 178 210	20 46 71 91 135 178	43 78 112 143 176 211	42 86 101 133 155 187	35 83 106 134 156 188
		237	233	217	234	234	228

176035	3	38 118 195	47 113 198	74 138 199	49 116 199	57 106 181	48 108 194
	5	36 73 118 142 212	51 93 139 184 220	36 73 136 187 222	54 96 141 187 221	51 93 137 185 222	64 109 136 171 213
	7	24 52 81 117 183 206	49 90 117 145 170 195	40 78 114 136 171 207	43 80 105 132 163 192	47 79 106 133 157 184	51 100 116 143 180 200
		215	224	231	224	219	223

225017	3	24 116 236	68 134 195	68 136 196	70 138 197	67 138 199	103 168 209
	5	23 72 154 201 229	21 76 128 162 216	25 75 108 142 213	21 76 137 166 211	27 78 131 169 215	33 83 135 177 208
	7	20 37 90 115 127 184	22 44 78 112 147 182	20 84 129 146 165 192	21 43 81 118 153 190	21 41 79 115 139 163	29 79 107 143 186 209
		218	219	233	223	204	236

241004	3	46 100 142	84 164 217	84 161 214	84 164 217	85 165 216	90 161 210
	5	28 84 135 167 225	47 102 158 183 218	43 82 111 155 216	50 105 162 195 225	44 100 144 166 218	61 110 161 199 229
	7	12 28 42 79 132 173	44 68 98 127 156 186	46 75 91 113 157 197	43 97 143 170 199 216	50 80 109 138 163 189	47 87 109 121 138 171
		196	219	227	232	220	212

385028	3	88 118 217	76 132 194	77 157 217	74 128 192	76 133 194	66 110 186
	5	44 93 135 169 219	56 93 133 173 214	56 119 165 198 231	54 90 119 156 210	58 98 136 175 215	45 86 133 169 221
	7	56 86 117 135 162 202	54 88 114 139 167 196	42 66 99 139 172 203	53 86 112 137 166 193	53 86 112 133 160 188	42 72 117 160 182 206
		226	226	231	225	222	224

388016	3	54 132 204	52 97 175	51 128 205	46 121 204	51 95 170	50 111 181
	5	56 104 148 204 246	49 91 133 176 214	41 97 120 159 217	49 91 138 182 217	50 90 135 182 215	30 68 88 136 210
	7	46 84 104 128 149 198	47 87 116 147 173 196	48 95 117 139 168 190	47 88 113 142 170 193	43 81 110 141 170 193	37 78 123 147 178 203
		220	224	221	224	222	233

2092	3	36 162 194	41 97 175	36 96 180	41 97 175	40 98 174	53 108 167
	5	34 62 120 212 248	31 61 94 127 181	30 62 92 119 181	32 63 92 121 174	30 62 96 127 175	31 74 97 128 179
	7	34 70 78 112 158 190	24 47 65 88 112 132	36 71 105 144 172 194	25 52 67 85 112 137	21 46 72 96 115 136	20 41 88 131 140 156
		227	185	217	189	174	202

14037	3	96 178 216	58 105 180	57 145 220	96 183 219	57 102 178	66 109 183
	5	44 92 148 184 216	60 109 148 187 221	56 105 156 202 229	56 104 148 189 223	55 99 144 188 222	48 95 141 185 221
	7	38 104 141 152 181 198	43 75 103 131 161 190	52 98 133 165 187 208	38 69 99 126 161 192	43 70 103 135 165 192	29 73 117 142 167 191
		223	223	232	224	224	222

55067	3	44 180 196	40 79 148	40 79 149	40 79 147	40 79 147	41 94 179
	5	33 63 84 118 164	38 63 99 135 170	39 84 119 159 203	37 63 100 137 172	38 62 98 135 173	37 81 100 137 177
	7	28 53 84 125 169 187	40 63 82 112 139 167	36 55 77 113 161 191	40 61 81 112 139 170	37 59 82 107 146 180	40 69 102 123 146 168
		237	200	206	205	200	201

169012	3	106 167 210	78 139 197	65 130 197	80 142 199	80 139 197	92 150 209
	5	25 36 59 80 143	55 100 137 180 220	51 87 122 165 216	52 98 136 177 218	59 103 143 187 222	63 117 152 175 219
	7	38 64 102 130 164 192	40 74 105 137 165 197	43 90 114 128 162 190	41 74 100 132 168 197	40 74 103 129 160 195	39 66 88 112 170 209
		219	229	223	227	226	232

The article "An Efficient Adaptive Salp Swarm Algorithm Using Type II Fuzzy Entropy for Multilevel Thresholding Image Segmentation" was published in 2022. Journal: Comput Math Methods Med.

**Table 4:** Parameters of TII-FE found by the proposed ECA and ASSA.

Im	PR	ASSA		HPFPPA-D		PSO		PFA		DE		PPA	
		*a*_*n*_	*c*_*n*_	*a*_*n*_	*c*_*n*_	*a*_*n*_	*c*_*n*_	*a*_*n*_	*c*_*n*_	*a*_*n*_	*c*_*n*_	*a*_*n*_	*c*_*n*_
41004	3	28 79 208	30 129 236	0 66 66	66 66 208	0 78 214	67 210 255	70138	69 138 248	0 70 130	70 130 240	2 81 95	69 91 209
	5	27 78 133 156	63 94 137 178	0 68 132 138	67 131 138 210	0 77 79 152	71 78 148 209	2 68 132 139	67 132 139 209	0 78 80 149	78 78 149 167	6 76 147 167	63 133 154
		242	252	210	255	215	255	210	254	167	250	219	215 252
	7	11 47 89 121	27 78 107 127	0 83 84 146	81 84 145 146	0 41 51 91	40 50 90 91	7 78 81 142	78 78 142 144	1 85 86 117	82 86 116 149	2 71 97 126	67 95 115 142
		142 177 229	173 228 245	146 210 210	209 210 255	91 178 178	178 178 255	144 211 212	208 211 255	150 161 212	159 212 255	142 174 211	170 201 244

176035	3	12 114 193	64 122 198	8 86 140	86 140 255	15 137 143	132 139 255	8 90 142	90 142 255	8 106 106	106 106 255	10 87 134	85 128 254
	5	31 61 112 123	42 86 124 162	9 93 93 184	93 93 184 184	8 65 85 186	64 81 186 187	12 95 96 186	95 96 185 187	10 93 93 182	92 93 181 188	22 108 113 158	106 110 158
		190	234	185	255	189	255	187	254	188	255	184	184 242
	7	18 45 71 102	30 59 92 132	9 89 90 144	89 90 144 145	16 65 91 136	64 91 136 136	8 79 81 129	78 80 128 135	15 79 79 132	78 79 132 133	10 92 109 124	92 108 122 162
		171 201 213	195 211 218	145 194 195	194 195 253	138 206 207	203 207 255	136 190 194	190 193 254	135 181 188	179 187 250	166 194 209	193 209 236

225017	3	20 46 231	28 186 242	1 134 134	134 134 255	1 36 136	135 136 255	1 138 138	138 138 255	134 143	134 142 255	45 167 170	160 169 248
	5	20 64 126 190	26 80 183 212	0 43 108 147	42 108 147 176	0 49 101 115	49 100 114 169	0 42 110 165	41 109 164 166	0 60 95 166	54 95 166 172	7 62 104 174	59 103 165 180
		215	244	177	255	170	255	166	255	174	255	181	234
	7	17 30 70 114	23 45 111 117	1 44 44 112	43 44 112 112	0 41 128 130	40 127 129 162	0 42 45 117	42 43 117 119	2 41 43 114	40 41 114 115	3 65 96 127	55 92 118 159
		120 175 206	134 193 230	112 181 183	181 182 255	162 172 211	168 211 255	120 188 191	185 191 255	115 162 163	162 163 245	175 196 224	196 222 248

241004	3	32 90 118	60 110 166	21 146 181	146 181 252	21 149 173	146 172 255	21 146 181	146 181 252	22 148 181	148 181 251	41 150 182	138 172 237
	5	20 65 124 150	36 103 147 185	22 72 133 183	71 132 183 183	21 65 105 134	64 98 117 175	22 77 132 192	77 132 191 198	22 68 134 153	66 132 153 179	31 98 128 195	91 121 193 202
		213	238	184	251	177	255	198	251	184	252	206	251
	7	8 24 30 61	16 32 55 97	21 68 68 127	67 68 127 127	21 71 80 103	71 79 102 123	22 66 130 158	64 128 156 181	23 78 81 138	77 81 137 138	26 72 105 115	67 101 113 127
		127 169 191	137 177 202	128 185 186	183 186 251	124 194 203	19,01,99,251	183 215 216	214 216 247	139 188 190	186 190 249	127 155 188	148 187 235

385028	3	81 115 182	95 121 252	19 132 132	132 132 255	18 136 179	135 177 255	19 128 129	128 128 255	18 133 133	133 133 255	31 102 122	101 117 250
	5	18 90 111 165	70 96 159 173	18 93 93 173	93 93 172 173	18 96 141 188	94 141 188 207	19 89 90 148	88 90 148 163	19 96 99 174	96 99 173 175	21 74 103 164	69 98 162 174
		201	238	173	255	207	255	165	254	175	255	190	252
	7	54 76 115 131	58 96 120 140	19 88 88 139	88 88 139 139	22 63 69 137	62 68 129 140	20 85 87 137	85 87 136 137	26 81 91 133	80 91 132 133	19 67 82 158	65 76 152 161
		161 189 220	163 216 233	139 195 197	195 196 254	142 202 206	201 203 255	140 192 195	192 194 254	134 187 189	186 188 254	162 205 209	202 206 239

388016	3	34 101 198	74 163 210	7 97 97	97 97 252	1,06,158	10,21,50,252	4 87 155	87 155,252	7 95 96	95 95 244	2 105 121	98 117 240
	5	43 98 138 204	69 110 158 205	7 90 91 176	90 91 174 176	0 91 104 138	81 103 136 179	7 90 93 182	90 91 182 182	10 90 90 182	89 90 179 182	5 61 75 107	55 74 101 165
		240	253	177	250	181	252	183	251	182	248	170	250
	7	30 80 98 113	62 88 110 143	7 87 87 145	86 87 144 149	3 94 95 139	93 95 139 139	9 86 90 136	85 89 135 147	7 80 85 136	78 81 135 145	5 71 108 139	69 85 137 155
		147 195 210	151 201 230	150 196 198	196 196 249	147 189 190	189 190 252	149 192 196	191 193 252	148 192 197	191 193 247	156 201 215	199 204 250

2092	3	12 134 184	59 190 204	0 82 111	82 111 238	0 77 118	72 115 241	0 82 111	82 111,239	0 80 116	79 115 231	13 97 119	93 118 214
	5	30 52 111 204	38 72 130 220	0 61 61 127	61 61 126 127	0 61 65 119	60 62 118 119	1 62 63 121	62 63 120 121	1 61 65 126	59 62 126 127	4 59 96 101	57 89 98 154
		245	251	127	235	120	241	122	226	129	221	155	202
	7	3 65 75 82	65 76 81 142	0 47 47 82 93	47 47 82 93	0 71 72 139	71 71 138 149	0 51 52 82 88	50 52 82 88 136	0 45 49 96 96	42 47 95 96	6 35 50 127	34 46 125 134
		146 178 225	170 202 229	132 133	131 132 237	150 194 195	194 194 239	137 138	137 240	136 136	134 136 212	135 145 167	144 167 237

14037	3	64 150 212	128 205 219	11 105 105	105 105 255	8 106 184	106 183 255	10 182 183	182 183 255	11 102 102	102 102 254	27 108 115	105 109 251
	5	40 74 126 180	48 110 170 188	11 109 109	109 109 186	8 104 110 201	104 106 201	11 103 189	101 105 189	12 98 101 188	97 100 187 188	15 86 114 178	81 104 168 192
		205	227	186 187	187 255	202	202 255	190	189 255	190	254	195	247
	7	33 80 138 150	43 128 144 154	11 74 76 131	74 75 130 131	11 94 102 165	92 101 164 165	11 64 74 123	64 73 123 129	17 68 73 134	68 72 133 136	13 49 100 134	45 96 133 149
		170 194 215	192 203 232	131 190 191	190 190 255	165 208 209	208 208 255	130 191 193	191 192 254	138 191 193	191 192 255	152 191 203	182 191 240

55067	3	24 176 191	64 184 201	13 73 84	66 84 211	13 75 83	67 82 215	13 73 85	66 84 209	13 74 84	66 83 210	19 63 143	62 125 214
	5	24 62 78 110	42 65 89 126	14 62 63 135	62 63 135 135	14 64 105 132	63 104 132 186	13 62 64 137	61 64 135 137	16 61 64 135	60 62 131 135	11 74 91 119	63 87 108 155
		133	195	135	205	186	220	139	204	135	211	159	195
	7	18 43 74 89	38 63 94 162	16 63 64 101	63 63 100 122	19 52 59 95	52 58 95 131	19 61 61 100	61 61 100 124	15 59 59 105	58 59 104 109	12 69 84 121	67 69 119 125
		166 176 223	173 199 251	124 154 181	153 180 219	132 190 191	190 191 220	125 152 189	152 188 220	112 180 180	179 180 219	136 158 188	155 177 214

169012	3	87 126 196	126 186 225	17 139 139	139 139 255	8 122 139	122 138 255	18 141 142	141 142 255	20 139 139	139 139 255	42 142 162	141 157 255
	5	24 32 45 80	27 40 74 81	9 100 100 175	100 100 174	15 87 89 155	87 87 154 175	8 96 100 173	95 99 172 181	14 103 103	103 103 183	28 100 138 167	97 134 165 183
		95	192	185	185 255	176	255	181	255	185 188	188 255	185	255
	7	15 50 82 119	61 78 122 141	8 72 76 135	71 76 134 139	11 74 106 122	74 106 122 133	9 72 76 125	72 76 123 139	8 73 76 129	72 74 129 129	24 64 69 110	54 67 107 114
		160 179 192	168 205 247	139 191 202	191 202 255	133 190 190	190 190 255	141 196 198	195 197 255	129 192 198	191 198 254	134 208 210	206 210 254

The article "An Efficient Adaptive Salp Swarm Algorithm Using Type II Fuzzy Entropy for Multilevel Thresholding Image Segmentation" was published in 2022. Journal: Comput Math Methods Med.

**Table 5:** Mean of objective function values attained by the proposed ASSA method for segmentation of digital images using TII-FE.

Im	PR	ASSA	HPFPPA-D	PSO	PFA	DE	PPA
41004	3	17.3864	17.3863	17.2156	17.2782	17.2791	16.9104
	5	24.2117	24.2115	23.9600	24.1390	24.0352	22.8482
	7	31.1427	31.1426	29.4424	30.9325	29.9948	28.8107

176035	3	17.7601	17.7601	17.5834	17.7495	17.7489	17.6123
	5	25.2170	25.2168	24.4512	25.1378	25.1447	24.2853
	7	31.3427	31.3426	30.5019	31.1211	30.8947	29.5311

225017	3	18.0951	18.0951	18.0792	18.0926	18.0747	17.4896
	5	24.8891	24.8890	24.5326	24.8027	24.6752	23.7939
	7	31.7468	31.7468	30.5922	31.5669	31.1628	29.1164

241004	3	17.8438	17.8439	17.3242	17.8300	17.8167	16.8263
	5	24.3558	24.3560	23.1237	24.1762	24.0404	23.4730
	7	30.5442	30.5444	29.6791	29.5852	30.0270	28.1811

385028	3	18.4241	18.4240	18.1789	18.4032	18.4061	17.8249
	5	25.0346	25.0345	24.6457	24.9557	24.9560	23.7739
	7	31.3952	31.3952	30.5094	31.1828	30.9945	29.1722

388016	3	17.7144	17.7143	17.3642	17.5825	17.6860	17.1471
	5	25.0007	25.0004	23.5646	24.9431	24.8289	23.3324
	7	31.1422	31.1422	30.5295	30.8938	30.5589	28.8578

2092	3	17.2421	17.2419	17.0647	17.2309	17.2207	16.8108
	5	24.0936	24.0933	23.8854	23.9760	23.8218	22.3837
	7	29.5949	29.5849	28.2241	29.3500	29.1886	27.3881

14037	3	18.0703	18.0702	17.6458	17.8294	18.0524	17.2870
	5	25.4902	25.4897	24.9791	25.3580	25.2849	23.4466
	7	31.5336	31.5335	30.9586	31.2953	31.1121	29.2095

55067	3	16.8166	16.8165	16.6824	16.7545	16.7693	15.8787
	5	23.0714	23.0715	22.1780	22.9317	22.8726	21.4793
	7	28.3676	28.3676	27.6598	28.1647	28.0640	26.3183

169012	3	18.3465	18.3464	18.2438	18.3321	18.3382	18.0177
	5	25.1464	25.1463	24.9975	25.1118	25.1026	24.4865
	7	31.4109	31.4109	31.0277	31.2431	31.2794	29.4929

The article "An Efficient Adaptive Salp Swarm Algorithm Using Type II Fuzzy Entropy for Multilevel Thresholding Image Segmentation" was published in 2022. Journal: Comput Math Methods Med.

**Table 6:** Comparison of the SSIM, MSE, and PSNR value of ASSA applied over benchmark images using the TII-FE.

Im	PR	MSE						PSNR						SSIM					
		ASSA	HPFPPA-D	PSO	PFA	DE	PPA	ASSA	HPFPPA-D	PSO	PFA	DE	PPA	ASSA	HPFPPA-D	PSO	PFA	DE	PPA
41004	3	3.55*E* + 02	3.56*E* + 02	4.06*E* + 02	3.83*E* + 02	3.63*E* + 02	5.75*E* + 02	2.27*E* + 01	2.26*E* + 01	2.20*E* + 01	2.23*E* + 01	2.25*E* + 01	2.05*E* + 01	8.76*E* − 01	8.76*E* − 01	8.70*E* − 01	8.73*E* − 01	8.74*E* − 01	8.61*E* − 01
	5	1.37*E* + 02	1.38*E* + 02	1.28*E* + 002	1.74*E* + 02	1.30*E* + 02	2.15*E* + 02	2.71*E* + 02	2.70*E* + 01	2.57*E* + 01	2.70*E* + 01	2.48*E* + 01	2.67*E* + 01	9.21*E* − 01	9.21*E* − 01	9.07*E* − 01	9.12*E* − 01	8.84*E* − 01	9.12*E* − 01
	7	8.69*E* + 01	8.71*E* + 01	1.02*E* + 02	1.05*E* + 02	8.91*E* + 01	1.17*E* + 02	2.92*E* + 01	2.87*E* + 01	2.79*E* + 01	2.86*E* + 01	2.80*E* + 01	2.74*E* + 01	9.23*E* − 01	9.22*E* − 01	9.15*E* − 01	9.22*E* − 01	9.22*E* − 01	9.13*E* − 01

176035	3	3.07*E* + 02	3.09*E* + 02	3.64*E* + 02	3.68*E* + 02	3.94*E* + 02	3.57*E* + 02	2.37*E* + 01	2.35*E* + 01	2.32*E* + 01	2.26*E* + 01	2.25*E* + 01	2.22*E* + 01	8.52*E* − 01	8.53*E* − 01	8.45*E* − 01	8.34*E* − 01	8.29*E* − 01	8.12*E* − 01
	5	1.28*E* + 02	1.30*E* + 02	1.69*E* + 02	1.32*E* + 02	1.30*E* + 02	1.89*E* + 02	2.72*E* + 01	2.70*E* + 01	2.59*E* + 01	2.69*E* + 01	2.70 + 01	2.54*E* + 01	8.71*E* − 01	8.71*E* − 01	8.57*E* − 01	8.70*E* − 01	8.71*E* − 01	8.53*E* − 01
	7	8.03*E* + 01	8.04*E* + 01	8.25*E* + 01	1.00*E* + 02	8.16*E* + 01	1.29*E* + 02	2.91*E* + 01	2.91*E* + 01	2.81*E* + 01	2.90*E* + 01	2.90*E* + 01	2.70*E* + 01	8.98*E* − 01	8.98*E* − 01	8.84*E* − 01	8.95*E* − 01	8.94*E* − 01	8.76*E* − 01

225017	3	3.30*E* + 02	3.31*E* + 02	3.19*E* + 02	3.27*E* + 02	3.41*E* + 02	3.51*E* + 02	2.31*E* + 01	2.31*E* + 01	2.30*E* + 01	2.28*E* + 01	2.27*E* + 01	2.29*E* + 01	8.47*E* − 01	8.48*E* − 01	8.45*E* − 01	8.39*E* − 01	8.36*E* − 01	8.44*E* − 01
	5	1.41*E* + 02	1.43*E* + 02	1.59*E* + 02	1.71*E* + 02	1.49*E* + 02	1.79*E* + 02	2.67*E* + 01	2.66*E* + 01	2.58*E* + 01	2.64*E* + 01	2.61*E* + 01	2.56*E* + 01	9.01*E* − 01	9.01*E* − 01	8.91*E* − 01	9.00*E* − 01	8.97*E* − 01	8.75*E* − 01
	7	8.87*E* + 01	8.89*E* + 01	9.53*E* + 01	1.09*E* + 02	8.94*E* + 01	1.25*E* + 02	2.86*E* + 01	2.86*E* + 01	2.78*E* + 01	2.86*E* + 01	2.83*E* + 01	2.72*E* + 01	9.23*E* − 01	9.22*E* − 01	9.16*E* − 01	9.22*E* − 01	9.21*E* − 01	9.16*E* − 01

241004	3	2.13*E* + 02	2.15 + 02	2.18*E* + 02	2.18*E* + 02	2.19*E* + 02	2.17*E* + 02	2.49*E* + 02	2.47*E* + 01	2.48*E* + 01	2.48*E* + 01	2.48*E* + 01	2.47*E* + 01	8.97*E* − 01	8.97*E* − 01	8.97*E* − 01	8.96*E* − 01	8.96*E* − 01	8.95*E* − 01
	5	1.39*E* + 02	1.40*E* + 02	1.78*E* + 02	1.88*E* + 02	1.95*E* + 02	1.74*E* + 02	2.57*E* + 01	2.54*E* + 01	2.67*E* + 01	2.57*E* + 01	2.56*E* + 01	2.52*E* + 01	8.91*E* − 01	8.91*E* − 01	8.71*E* − 01	8.87*E* − 01	8.83*E* − 01	8.80*E* − 01
	7	7.78*E* + 01	7.79*E* + 01	1.01*E* + 02	8.68*E* + 01	9.55*E* + 01	1.35*E* + 02	2.95*E* + 01	2.92*E* + 01	2.83*E* + 01	2.81*E* + 01	2.87*E* + 01	2.68*E* + 01	9.29*E* − 01	9.30*E* − 01	9.20*E* − 01	9.15*E* − 01	9.21*E* − 01	8.92*E* − 01

385028	3	3.18*E* + 02	3.19*E* + 02	3.29*E* + 02	3.28*E* + 02	3.32*E* + 02	3.20*E* + 02	2.42*E* + 01	2.40*E* + 01	2.31*E* + 01	2.30*E* + 01	2.31*E* + 01	2.29*E* + 01	7.85*E* − 01	7.86*E* − 01	7.82*E* − 01	7.67*E* − 01	7.69*E* − 01	7.62*E* − 01
	5	1.25*E* + 02	1.26*E* + 02	1.76*E* + 02	1.41*E* + 02	1.38*E* + 02	2.08*E* + 02	2.71*E* + 01	2.71*E* + 01	2.57*E* + 01	2.66*E* + 01	2.67*E* + 01	2.49*E* + 01	8.69*E* − 01	8.68*E* − 01	8.44*E* − 01	8.46*E* − 01	8.48*E* − 01	8.17*E* − 01
	7	7.14*E* + 01	7.15*E* + 01	7.27*E* + 01	7.57*E* + 01	7.25*E* + 01	1.02*E* + 02	2.99*E* + 01	2.96*E* + 01	2.93*E* + 01	2.95*E* + 01	2.95*E* + 01	2.81*E* + 01	9.07*E* − 01	9.07*E* − 01	9.02*E* − 01	9.06*E* − 01	9.03*E* − 01	8.74*E* − 01

388016	3	3.51*E* + 01	3.54*E* + 02	5.32*E* + 02	3.76*E* + 02	5.49*E* + 02	3.60*E* + 02	2.11*E* + 01	2.09*E* + 01	2.26*E* + 01	2.24*E* + 01	2.26*E* + 01	2.07*E* + 01	7.47*E* − 01	7.44*E* − 01	7.39*E* − 01	7.33*E* − 01	7.38*E* − 01	6.89*E* − 01
	5	1.43*E* + 01	1.46*E* + 02	1.51*E* + 02	1.53*E* + 02	2.13*E* + 02	1.49*E* + 02	2.68*E* + 01	2.66*E* + 01	2.65*E* + 01	2.64*E* + 01	2.63*E* + 01	2.48*E* + 01	8.29*E* − 01	8.29*E* − 01	8.25*E* − 01	8.21*E* − 01	8.20*E* − 01	7.94*E* − 01
	7	8.02*E* + 02	8.04*E* + 01	8.25*E* + 01	8.35*E* + 01	8.19*E* + 01	8.88*E* + 01	2.92*E* + 01	2.91*E* + 01	2.89*E* + 01	2.90*E* + 01	2.90*E* + 01	2.86*E* + 01	8.81*E* − 01	8.82*E* − 01	8.72*E* − 01	8.78*E* − 01	8.77*E* − 01	8.70*E* − 01

2092	3	3.03*E* + 01	3.06*E* + 02	3.10*E* + 02	3.15*E* + 02	3.48*E* + 02	3.10*E* + 02	2.32*E* + 01	2.31*E* + 01	2.33*E* + 01	2.32*E* + 01	2.32*E* + 01	2.27*E* + 01	8.83*E* − 01	8.82*E* − 01	8.82*E* − 01	8.82*E* − 01	8.82*E* − 01	8.79*E* − 01
	5	1.28*E* + 02	1.32*E* + 02	1.51*E* + 02	1.48*E* + 02	1.55*E* + 02	1.80*E* + 02	2.71*E* + 01	2.69*E* + 01	2.64*E* + 01	2.62*E* + 01	2.63*E* + 01	2.56*E* + 01	9.22*E* − 01	9.22*E* − 01	9.22*E* − 01	9.17*E* − 01	9.20*E* − 01	9.14*E* − 01
	7	6.89*E* + 01	7.00*E* + 01	8.19*E* + 01	8.37*E* + 01	7.03*E* + 01	9.61*E* + 01	2.96*E* + 01	2.97*E* + 01	2.89*E* + 01	2.97*E* + 01	2.90*E* + 01	2.83*E* + 01	9.52*E* − 01	9.52*E* − 01	9.28*E* − 01	9.51*E* − 01	9.46*E* − 01	9.20*E* − 01

14037	3	3.12*E* + 01	3.13*E* + 02	3.58*E* + 02	3.51*E* + 02	9.28*E* + 02	3.47*E* + 02	2.38*E* + 01	2.36*E* + 01	2.32*E* + 01	2.27*E* + 01	2.27*E* + 01	1.85*E* + 01	8.11*E* − 01	8.11*E* − 01	8.03*E* − 01	7.92*E* − 01	7.99*E* − 01	7.15*E* − 01
	5	2.10*E* + 01	2.12*E* + 02	2.23*E* + 02	2.32*E* + 02	2.20*E* + 02	2.41*E* + 02	2.49*E* + 01	2.49*E* + 01	2.45*E* + 01	2.47*E* + 01	2.47*E* + 01	2.43*E* + 01	8.36*E* − 01	8.38*E* − 01	8.09*E* − 01	8.21*E* − 01	8.13*E* − 01	8.02*E* − 01
	7	7.28*E* + 02	7.31*E* + 01	8.78*E* + 01	9.31*E* + 01	8.33*E* + 01	1.70*E* + 02	2.94*E* + 01	2.95*E* + 01	2.84*E* + 01	2.89*E* + 01	2.87*E* + 01	2.58*E* + 01	8.97*E* − 01	8.97*E* − 01	8.75*E* − 01	8.86*E* − 01	8.77*E* − 01	8.36*E* − 01

55067	3	3.75*E* + 01	3.76*E* + 02	3.87*E* + 02	3.84*E* + 02	3.84*E* + 02	4.07*E* + 02	2.26*E* + 01	2.24*E* + 01	2.23*E* + 01	2.23*E* + 01	2.23*E* + 01	2.20*E* + 01	9.45*E* − 01	9.44*E* − 01	9.41*E* − 01	9.42*E* − 01	9.44*E* − 01	9.41*E* − 01
	5	8.85*E* + 02	8.88*E* + 01	1.10*E* + 02	1.10*E* + 02	1.08*E* + 02	1.18*E* + 02	2.88*E* + 01	2.86*E* + 01	2.77*E* + 01	2.78*E* + 01	2.77*E* + 01	2.74*E* + 01	9.61*E* − 01	9.63*E* − 01	9.52*E* − 01	9.60*E* − 01	9.60*E* − 01	9.36*E* − 01
	7	4.24*E* + 02	4.26*E* + 01	4.66*E* + 01	5.30*E* + 01	4.53*E* + 01	6.91*E* + 01	3.19*E* + 01	3.18*E* + 01	3.09*E* + 01	3.16*E* + 01	3.14*E* + 01	2.97*E* + 01	9.67*E* − 01	9.67*E* − 01	9.59*E* − 01	9.61*E* − 01	9.60*E* − 01	9.57*E* − 01

169012	3	2.69*E* + 01	2.72*E* + 02	3.01*E* + 02	2.79*E* + 02	2.75*E* + 02	3.10*E* + 02	2.41*E* + 01	2.38*E* + 01	2.33*E* + 01	2.37*E* + 01	2.37*E* + 01	2.32*E* + 01	8.05*E* − 01	8.05*E* − 01	7.83*E* − 01	8.03*E* − 01	8.05*E* − 01	7.75*E* − 01
	5	1.46*E* + 01	1.47*E* + 02	1.65*E* + 02	1.65*E* + 02	1.53*E* + 02	1.90*E* + 02	2.63*E* + 01	2.64*E* + 01	2.60*E* + 01	2.63*E* + 01	2.60*E* + 01	2.53*E* + 01	8.51*E* − 01	8.47*E* − 01	8.41*E* − 01	8.43*E* − 01	8.41*E* − 01	8.35*E* − 01
	7	8.44*E* + 02	8.45*E* + 01	1.02*E* + 02	8.58*E* + 01	8.57*E* + 01	1.26*E* + 02	2.88*E* + 01	2.89*E* + 01	2.80*E* + 01	2.88*E* + 01	2.88*E* + 01	2.71*E* + 01	8.92*E* − 01	8.91*E* − 01	8.81*E* − 01	8.90*E* − 01	8.91*E* − 01	8.66*E* − 01

The article "An Efficient Adaptive Salp Swarm Algorithm Using Type II Fuzzy Entropy for Multilevel Thresholding Image Segmentation" was published in 2022. Journal: Comput Math Methods Med.

## Data Availability

The data that support the findings of this study are available on request from the corresponding author.
